RETRACTED

# Silencing of LncRNA PVT1 inhibits the proliferation, migration and fibrosis of high glucose-induced mouse mesangial cells via targeting microRNA-93-5p

**DOI:** 10.1042/BSR20194427

**Published:** 2020-05-04

**Authors:** Jianzhou Li, Qing Zhao, Xiaohong Jin, Yanhua Li, Jian Song

**Affiliations:** 1 Department of Endocrinology, Caoxian People’s Hospital, East Qinghe Road, South Fumin Avenue, Caoxian Development Zone, Heze City 274400, Shandong Province, China; 2 Department of Medical, First People’s Hospital of Jinan City, No. 132, Daminghu Road, Lixia District, Jinan City 250011, Shandong Province, China; 3 Department of Nephrology, Qilu Hospital of Shandong University, No. 107, Wenhua West Road, Jinan City 250012, Shandong Province, China

**Keywords:** diabetic nephropathy, LncRNA-PVT1, miR-93-5p, mouse mesangial cells, PI3K/Akt/mTOR pathway

## Abstract

**Objective:** The present study aimed to investigate the regulatory role of long non-coding RNA plasmacytoma variant translocation 1 (PVT1) on high glucose (HG)-induced mouse mesangial cells (MMCs).

**Methods:** PVT1 expression in diabetic nephropathy (DN) mice and HG-induced MMCs was detected by qRT-PCR. EdU and Colony formation, Annexin V-PI staining, Muse cell cycle, Scratch, and Transwell assays were performed to detect the cell proliferation, apoptosis, cell cycle, migration, and invasion, respectively. The contents of fibrosis factors in cell-culture supernatants were detected by enzyme-linked immunosorbent assay (ELISA). Western blot was performed to detect the expression of factors involved in apoptosis, cell cycle, migration and invasion, fibrosis, and PI3K/Akt/mTOR pathway. The targeting relation between miR-93-5p and PVT1 was predicted by StarBase3.0 (an online software for analyzing the targeting relationship) and identified by Dual-luciferase reporter (DLR) assay.

**Results:** PVT1 was overexpressed in DN kidney tissues and HG-induced MMCs. HG-induced MMCs exhibited significantly increased EdU-positive cells, cell colonies, S and G_2_/M phase cells, migration and invasion ability, and contents of fibrosis factors, as well as significantly decreased apoptosis rate compared with NG-induced MMCs. HG significantly up-regulated Bcl-2, CyclinD1, CDK4, N-cadherin, vimentin, Col. IV, FN, TGF-β1 and PAI-1, and down-regulated Bax, cleaved caspase-3, cleaved PARP, and E-cadherin in MMCs. Silencing of PVT1 eliminated the effects of HG in MMCs and blocked PI3K/Akt/mTOR pathway. MiR-93-5p was a target of PVT1, which eliminated the effects of PVT1 on HG-induced MMCs.

**Conclusions:** PVT1 silencing inhibited the proliferation, migration, invasion and fibrosis, promoted the apoptosis, and blocked PI3K/Akt/mTOR pathway in HG-induced MMCs via up-regulating miR-93-5p.

RETRACTED

## Introduction

Diabetic nephropathy (DN), characterized by decreased glomerular filtration, proteinuria, and renal fibrosis is a common diabetes-associated disease [1]. DN affects more than 40% diabetic patients worldwide, and leads to millions of deaths due to end-stage kidney disease [2]. The occurrence of DN has been attributed to diverse factors, such as hyperglycemia, accumulation of advanced glycosylation products, and activation of cytokines [3]. Although many attempts have been made to the clinical treatment of DN [4,5], the modern medical treatment is still unable to completely prevent the development and deterioration of DN due to the insufficient understanding of the pathological mechanisms involving DN [6].

Long non-coding RNAs (lncRNAs) are important transcripts that take part in the regulation of disease pathways [7–10]. The dysregulation of lncRNAs has been widely reported in various diseases, including DN [11,12]. LncRNA plasmacytoma variant translocation 1 (PVT1) is an important lncRNA regulator in diabetes [13]. It has been proved that autophagy ameliorates cognitive impairment in diabetic mice through activating PVT1 [14]. Type 1 diabetes-induced end-stage renal disease (ESRD) is closely associated with the variants in PVT1 [15]. PVT1 mediates the accumulation of extracellular matrix in DN [16]. LncRNAs can modulate the translation and degradation of mRNAs through interacting with microRNAs (miRs) [17]. The biological function of PTV1 during the disease process is realized by targeting specific miRs [18]. Six locations on PVT1 are revealed on miR-1204, -1205, -1206, 1207-3p, -1207-5p, and -1208 [19]. The mediation effect of PTV1 during extracellular matrix accumulation in kidney cells of DN is realized by targeting miR-1207-5p [20]. MiR-93 is an onco-miR in cancer [21], that is also a regulator in DN [22]. It has been proved that the serum miR-93 is low-expressed in DN patients [23]. Comparative miR expression profile arrays showed that miR-93 is a signature miR in hyperglycemic condition [24]. Up-regulation of miR-93 inhibits epithelial–mesenchymal transformation and renal fibrogenesis in TGF-β1-induced HK2 cells [25]. Although the biological functions of PTV1 and miR-93 in DN have been mentioned by previous studies, the detailed molecular mechanism of PTV1 involving miR-93 in DN remains unclear.

In the present study, the regulatory role of PVT1 on the proliferation, apoptosis, cell cycle, migration, invasion, and fibrosis of high glucose (HG)-induced mouse mesangial cells (MMCs) was evaluated. The regulatory mechanism of PVT1 involving miR-93 was analyzed. The present study may lay a novel theoretical basis for the treatment of DN.

RETRACTED

## Methods

### Animals

The db/bd mouse is a well-established animal model of type II diabetes. A total of ten SPF db/db mice (SPF grade, 4-week-old, Strain: BKS.Cg-+Leprdb/+Leprdb/J, 20–30 g) and ten non-diabetic db/m mice (SPF grade, 4-week-old, Strain: BKS.Cg-Dock7m+/+Leprdb/J, 20–30 g) were obtained from the Model Animal Research Center of Nanjing University (Nanjing, China). Mice were fed in a standalone environment at 22°C and 50% relative humidity under an artificial cycle of 12-h day and 12-h night. After 4 days of feeding with standard diet (12% fat, 28% protein, and 60% carbohydrates, SLAC, Shanghai, China) for acclimatization, mice were anesthetized by intraperitoneal injection of 50 mg/kg sodium pentobarbital, and killed by cervical dislocation. The kidney tissues were then stripped and used for detecting the expression of PVT1 by *qRT-PCR*. The present study was approved by the local ethics committee of our hospital. All animal experiments were performed in the Experimental Animal Center of Qilu Hospital of Shandong University in accordance with the care and use of laboratory animals (National Institutes of Health, U.S.A.).

### Cell culture

MMCs (SV40 MES13, established from the kidney of a mouse transgenic for the SV40 early region) were purchased from the Cell Bank of the Chinese Academy of Sciences (Shanghai, China). MMCs were cultured in a mixture of DMEM containing 10% FBS and Ham’s F12 medium (3:1) containing 14 mM HEPES, and maintained in a humidified incubator (MCO-15AC, SANYO) with 5% CO_2_ at 37°C. The medium was refreshed every 48 h, and cells were passaged at 80% confluence. Logarithmic growth phase cells at the third passage were used for transfection.

### Cell treatment and transfection

PVT1 siRNA (si-PVT1) and siRNA negative control (si-NC) were synthesized by Shenggong Bioengineering Co., Ltd. (Shanghai, China) (Table 1). MiR-93-5p mimics, miR-93-5p inhibitor, mimics negative control (mimics-NC), and inhibitor negative control (INC) were purchased from Jima Pharmaceutical Technology Co., Ltd. (Shanghai, China). Cells were transfected with the above agents by using a Lipofectamine kit (Invitrogen). Cells without transfection were considered as the control. The transfection efficiency was identified by qRT-PCR. After the transfection for 48 h, cells were incubated in DMEM containing 5.55 mmol/l (normal physiological environment, NG group) or 30 mmol/l d-Glucose (diabetic physiological environment, HG group) for another 48 h. Cells were collected for the following assay.

**Table 1:** The sequences of siRNAs and primers

Primer	Sequence
siPVT1	Forward: 5′-GCUUGGAGGCUGAGGAGUUTT-3′
	Reverse: 5′-AACUCCUCAGCCUCCAAGCTT-3′
siNC	Forward: 5′-UUCUCCGAACGUGUCACGUTT-3′
	Reverse: 5′-ACGUGACACGUUCGGAGAATT-3′
LncRNA-PVT1	Forward: 5′-ATTGAGATGTGAAGCGTTGA-3′
	Reverse: 5′-AGGCACCTTTCCCAGTT-3′
CyclinD1	Forward: 5′-AGCTCCTGTGCTGCGAAGTGGA-3′
	Reverse: 5′-AGTGTTCAATGAAATCGTGCGGG-3′
CDK4	Forward: 5′-AGTAATGGGACCGTCAAGC-3′
	Reverse: 5′-CACCAAGACTGGGAAAGG-3′
*miR-93-5P*	Forward: 5′-AGGCCCAAAGTGCTGTTCGT-3′
	Reverse: 5′-GTGCAGGGTCCGAGG-3′
U6	Forward: 5′-CTCGCTTCGGCAGCACA-3′
	Reverse: 5′-AACGCTTCACGAATTTGCGT-3′
GAPDH	Forward: 5′-TGACGTGCCGCCTGGAGAAAC-3′
	Reverse: 5′-CCGGCATCGAAGGTGGAAGAG-3′

RETRACTED

### qRT-PCR

Total RNA was extracted from kidney tissues and MMCs by using TRIzol reagent (Invitrogen), and then reverse-transcribed on a SimpliAmp PCR instrument (Applied Biosystems, Foster City, CA, U.S.A.). The qRT-PCR was performed on an ABI7500 Sequence Detection System (Applied Biosystems). The PCR program included 40 cycles of 95°C for 10 min, 95°C for 10 s, 60°C for 20 s, and 72°C for 34 s. The relative mRNA expression level was analyzed by the 2^−ΔΔ*C*_t_^ method [26]. Oligonucleotide primers were synthesized by Biotechnology Bioengineering Co., Ltd. (Shanghai, China), and the primer sequences were shown in Table 1.

### Western blot

Total proteins were extracted from cells using lysis buffer, and quantified using a BCA kit (Invitrogen). Then, 20 μg protein samples were run in 10% SDS/PAGE, and transferred on to PVDF membrane. Afterward, the membrane was blocked with 5% skim milk in TBST solution for 2 h, and incubated with primary antibody overnight at 4°C. The antibodies included E-cadherin (1:1000, 3195, CST), N-cadherin (1:1000,13116, CST), Vimentin (1:1000, 5741, CST), GAPDH (1:1000, 5174, CST), Col. IV (1:10000, ab6586, Abcam), FN (1:10000, ab2413, Abcam), TGF-β1 (1:10000, ab92486, Abcam), PAI-1 (1:10000, ab66705, Abcam), Bcl-2 (1:1000, ab196495, Abcam), Bax (1:1000, ab199677, Abcam), cleaved caspase-3 (1:1000, ab49822, Abcam), cleaved PARP (1:1000, ab32064, Abcam), CyclinD1 (1:5000, ab226977, Abcam), CDK4 (1:3000, ab137675, Abcam), PI3K (1:1000, 4292, CST), p-PI3K (1:1000, 4228, CST), Akt (1:1000, 9272, CST), p-Akt (1:1000, 4060, CST), mTOR (1:1000, 2972, CST), and p-mTOR (1:1000, 2971, CST). GAPDH was used as the internal control. After three washings with TBST, the membrane was incubated with HRP-labeled secondary antibody (1:1000, Sigma) for 2 h at 25°C. An enhanced chemiluminescence Plus (Thermo Fisher) was used to visualize the protein bands. The gray value was measured by using a Lab Works 4.5 software. Western blot was performed in three independent repetitions, and the representative images were shown.

### EdU and colony formation assay

An EdU cell proliferation detection kit (Ruibo Biotechnology Co., Ltd., Guangzhou, China) was used for EdU assay (cell proliferation). Briefly, cells were labeled with EdU, fixed with 4% paraformaldehyde, and then stained with DAPI. The EdU fluorescence (red) was detected by a Nikon A1R laser scanning confocal microscope (NIKON, Tokyo, Japan).

RETRACTED

For Colony formation assay, cells were seeded into six-well plates (300 cells/well) and cultured for 2 weeks. Cells were then fixed with 4% paraformaldehyde for 10 min and stained with Crystal Violet for 15 min. The stained colonies were observed under an inverted microscope (Olympus Ckx53, Japan), and counted using ImageJ (1.48 V) software.

### Annexin V-PI assay

An Annexin V-PI kit (Invitrogen) was used for the detection of cell apoptosis. Briefly, cells were stained with Annexin V-EGFP and PI for 15 min under darkness at 25°C. The apoptosis rate was then analyzed on a Muse™ cytometer (EMD Millipore, U.S.A.).

### Cell cycle analysis

A Muse™ Cell Cycle Reagent (Invitrogen) was used for the detection of cell cycle. Briefly, cells were fixed in 70% ethanol, and incubated with Muse™ Reagent in the dark for 30 min at 25°C. The cell cycle was then analyzed on a Muse™ cytometer (EMD Millipore).

### Scratch assay

Cells were seeded into six-well plate, and cultured in serum-free DMEM until 90% confluence. A scratch wound was then made in each well with a pipet tip. Cell debris was removed by washing with PBS. After 48 h of culturing in serum-free DMEM, the scratch width was photographed under an inverted microscope (Olympus Ckx53). The migration rate = (1 − scratch width at measurement/initial scratch width) × 100%.

### Transwell assay

The cell invasion was detected by using transwell chambers (Corning Corporation, Midland, MI, U.S.A.). Briefly, cells were seeded into Matrigel-coated upper chamber. The lower chamber was filled with DMEM. After 48 h of incubation, cells on the lower chamber were fixed with 4% paraformaldehyde for 15 min and stained with 0.1% Crystal Violet for 20 min. The stained cells were observed under an inverted microscope (Olympus Ckx53), and counted randomly at five fields of views at 200× magnifications.

### Enzyme-linked immunosorbent assay for fibrosis factors

Cells were cultured for 48 h after transfection, and the cell-culture supernatants were collected. The contents of Col. IV, PAI-1, FN, and TGF-β1 in the supernatants were detected by using enzyme-linked immunosorbent assay (ELISA) kits (BioSource International, Camarillo, CA, U.S.A.) in accordance with the manufacturer’s instructions.

### Dual-luciferase reporter gene assay

The binging site of PVT1 in miR-93-5p was predicted by StarBase3.0 (an online software for analyzing the targeting relationship). A Dual-luciferase reporter gene (DLR) kit (Promega, U.S.A.) was used to identify the relationship between PVT1 and miR-93-5p. The mutant sequence (MT) and the wild sequence (WT) of PVT1 were amplified according to the binging sequences, and then cloned into the pmirGLO luciferase vector. HEK-293T cells were then co-transfected with WT/MT and miR-93-5p mimics/miR-93-5p mimics NC (Shanghai Jima Pharmaceutical Technology Co., Ltd.), and grouped as MT + mimics, MT + NC, WT + mimics, and WT + NC group. After 48 h of transfection, the fluorescence was measured on a Microplate Reader (Invitrogen).

RETRACTED

### Statistical analysis

All assays were performed in triplicate. Data were expressed as mean ± standard deviation (SD). All statistical analyses were performed by SPSS 20.0 and GraphPad.Prism 5.01 statistical software. The homogeneity of variances was tested using Levene test. Data that passed Levene test were further analyzed using one-way ANOVA, followed by Tukey’s test (between two groups). *P*<0.05 represented statistically significant at the 5% level, *P*<0.01 represented statistically significant at the 1% level, and *P*<0.001 represented statistically significant at the 0.1% level.

## Results

### PVT1 was up-regulated in DN mice and HG-induced MMCs

The expression of PVT1 was detected in kidney tissues of DN mice and HG-induced MMCs by qRT-PCR. PVT1 expression was significantly higher in kidney tissues of db/db mice (DN) than those in tissues of db/m mice (Normal) (*P*<0.001) (Figure 1A). In addition, PVT1 was significantly up-regulated in HG-induced MMCs compared with NG-induced MMCs (*P*<0.001) (Figure 1B).

**Figure 1:** Expression of LncRNA-PVT1 in kidney tissues and MMCs (**A**) qRT-PCR was used to detect the expression of LncRNA-PVT1 in kidney tissues of db/m (Normal) and db/db (DN) mice; ***, *P*<0.001 compared with the db/m mice. (**B**) qRT-PCR was used to detect the expression of LncRNA-PVT1 in MMCs under normal glucose (NG) and HG conditions; ***, *P*<0.001 compared with the NG group.

### Silencing of PVT1 inhibited the proliferation of HG-induced MMCs

PVT1 was silenced in HG-induced MMCs by the transfection of PVT1 siRNA (siPVT1). The mRNA expression of PVT1 in the HG + siPVT1 group was significantly lower than that in the HG group (*P*<0.001). The expression of PVT1 was not significantly different between the HG group and the HG + siNC group (Figure 2A). EdU assay showed that the percentage of EdU cells in the HG group was significantly higher than that in the NG group (*P*<0.001). The percentage of EdU cells was significantly decreased in the HG + siPVT1 group compared with that in the HG group (*P*<0.001) (Figure 2B). Colony formation assay showed consistent results with EdU assay (all *P*<0.001) (Figure 2C). In addition, the cell apoptosis was opposite to the cell proliferation detected above (all *P*<0.001) (Figure 2D). The expression of Bax, cleaved caspase-3, and cleaved PARP in the HG group was significantly lower than that in the NG group (all *P*<0.001). The expression of Bax, caspase-3, and PARP was significantly increased in the HG + siPVT1 group compared with that in the HG group (all *P*<0.05). The expression change of Bcl-2 was opposite to that of Bax (all *P*<0.001) (Figure 2E).

RETRACTED

**Figure 2:** Effects of lncRNA-PVT1 on the proliferation and apoptosis of MMCs under HG condition (**A**) RNA interference efficiency; ***, *P*<0.001 compared with the HG group. (**B**) EdU assay was used to detect the proliferation ability (×200). (**C**) Colony formation assay was used to detect the colony forming ability. (**D**) Flow cytometry was used to detect the apoptosis rate. (**E**) Western blot was used to detect the expression of apoptotic proteins (Bcl-2, Bax, cleaved caspase-3, cleaved PARP). ***, *P*<0.001 compared with NG group; ^#^, *P*<0.05, ^##^, *P*<0.01, ^###^, *P*<0.001 compared with the HG group. The data among multigroups were analyzed by one-way ANOVA, followed by Tukey’s test (between two groups).

### Silencing of PVT1 influenced the cell cycle of HG-induced MMCs

The percentages of cells in S and G_2_/M phase were significantly higher and the percentage of cells in G_0_/G_1_ phase was significantly lower in the HG group than that in the NG group (all *P*<0.001). The transfection of siPVT1 eliminated the effects of HG on the cell cycle of MMCs (all *P*<0.001), suggesting that PVT1 silencing might block the cell cycle of HG-induced MMCs in G_0_/G_1_ phase (Figure 3A,B). The expression of Cyclin D1 and CDK4 in HG-induced MMCs was further detected by qRT-PCR and Western blot. CyclinD1 and CDK4 in the HG group were significantly up-regulated compared with the NG group at both the mRNA and protein level (all *P*<0.001). The mRNA and protein expression of CyclinD1 and CDK4 were decreased in the HG + siPVT1 group compared with those in the HG group (all *P*<0.001) (Figure 3C–E).

**Figure 3:** Effect of lncRNA-PVT1 on the cell cycle of MMCs under HG condition (**A**) Flow cytometry was used to detect the cell cycle. (**B**) The percentages of cells in different cell cycle phases. (**C**) qRT-PCR was used to detect the expression of CyclinD1. (**D**) qRT-PCR was used to detect the expression of CDK4. (**E**) Western blot was used to detect the expression of CyclinD1 and CDK4. ***, *P*<0.001 compared with the NG group; ^###^, *P*<0.001 compared with the HG group. The data among multigroups were analyzed by one-way ANOVA, followed by Tukey’s test (between two groups).

RETRACTED

### Silencing of PVT1 inhibited the migration and invasion of HG-induced MMCs

Scratch and Transwell assays showed that the cell migration and invasion ability were significantly enhanced in the HG group compared with the NG group (all *P*<0.01). The transfection of siPVT1 inhibited the migration and invasion ability of HG-induced MMCs (all *P*<0.05) (Figure 4A,B). Western blot showed that the expression of E-cadherin was significantly lower, and the expression of N-cadherin and vimentin was significantly higher in the HG group than that in the NG group (all *P*<0.001). The transfection of siPVT1 significantly reversed the expression of E-cadherin, N-cadherin, and vimentin in HG-induced MMCs (all *P*<0.01) (Figure 4C).

**Figure 4:** Effects of lncRNA-PVT1 on the migration and invasion of MMCs under HG condition (**A**) Scratch assay was used to detect the migration ability (×200). (**B**) Transwell assay was used to detect the invasion ability (×200). (**C**) Western blot was used to detect the expression of EMT proteins (N-cadherin, vimentin, and E-cadherin). **, *P*<0.01, ***, *P*<0.001 compared with the NG group; ^#^, *P*<0.05, ^##^, *P*<0.01, ^###^, *P*<0.001 compared with the HG group. The data among multigroups were analyzed by one-way ANOVA, followed by Tukey’s test (between two groups).

### Silencing of PVT1 inhibited the fibrosis of HG-induced MMCs

The contents of fibrosis factors in the supernatant of MMCs were detected by ELISA. The contents of Col. IV, FN, TGF-β1, and PAI-1 in the HG group were significantly higher than those in the NG group (all *P*<0.001). The contents of fibrosis factors in the HG+siPVT1 group were significantly decreased compared with those in the HG group (all *P*<0.01) (Figure 5A–D). In addition, Western blot showed that the expression of fibrosis factors was consistent with the ELISA results (all *P*<0.01) (Figure 5E).

**Figure 5:** Effect of lncRNA-PVT1 on the fibrosis of MMCs under HG condition (**A–D**) ELISA was used to detect the contents of fibrosis proteins (Col. IV, FN, TGF-β1, and PAI-1). (**E**) Western blot was used to detect the expression of fibrosis proteins. ***, *P*<0.001 compared with the NG group; ^##^, *P*<0.01, ^###^, *P*<0.001 compared with the HG group. The data among multigroups were analyzed by one-way ANOVA, followed by Tukey’s test (between two groups).

### MiR-93-5p was the target gene of PVT1

A binging site of PVT1 at miR-93-5p was predicted by StarBase3.0 software (Figure 6A). Because miR-93 plays an important role in the progression of DN, the targeting relation between miR-93-5p and PVT1 was further analyzed. DLR assay showed that the luciferase activity in the WT + mimics group was significantly lower than that in the WT + NC group (*P*<0.001) (Figure 6B). The mRNA expression of PVT1 was significantly higher in the inhibitor group and significantly lower in the mimics group than that in the Mock group (all *P*<0.001). The expression of PVT1 was not significantly influenced by the transfection of mimics-NC and INC. In addition, the expression of miR-93-5p in the HG group was significantly lower than that in the NG group (*P*<0.001). The transfection of siPVT1 significantly up-regulated miR-93-5p in HG-induced MMCs (*P*<0.001) (Figure 6C,D).

RETRACTED

**Figure 6:** MiR-93-5p was the target gene of LncRNA-PVT1 (**A**) StarBase3.0 software was used to predict the binding site of miR-93-5p to PVT1. (**B**) Dual luciferase reporter gene assay was used to identify the relationship between miR-93-5p and PVT1; ***, *P*<0.001 compared with the WT + NC group. (**C**) qRT-PCR was used to detect the expression of PVT1 in cells transfected with miR-93-5p mimics or inhibitor; ***, *P*<0.001 compared with the Mock group; ^###^, *P*<0.001 compared with the Mock group. (**D**) qRT-PCR was used to detect the expression of miR-93-5p in cells transfected with siPVT1; ***, *P*<0.001 compared with the NG group; ^###^, *P*<0.001 compared with the HG group. The data among multigroups were analyzed by one-way ANOVA, followed by Tukey’s test (between two groups).

### MiR-93-5p eliminated the role of PVT1 in HG-induced MMCs

MiR-93-5p inhibitor was used to silence miR-93-5p in HG-induced MMCs. The mRNA expression of miR-93-5p in the inhibitor group was significantly down-regulated compared with that in the Mock group (*P*<0.001). The expression of miR-93-5p was not significantly different between the INC group and the Mock group (Figure 7A). The miR-93-5p inhibitor and siPVT1 were then con-transfected into HG-induced MMCs. The cell proliferation, migration, invasion, and fibrosis ability were promoted by the transfection of miR-93-5p inhibitor, and inhibited by the transfection of siPVT1 (all *P*<0.05). The transfection of miR-93-5p inhibitor significantly eliminated the effects of siPVT1 on the above biological processes of HG-induced MMCs (all *P*<0.05) (Figure 7B–E).

**Figure 7:** MiR-93-5p eliminated the effect of LncRNA-PVT1 in MMCs under HG condition (**A**) The transfection efficiency of miR-93-5p inhibitor; ***, *P*<0.001 compared with the Mock group. (**B**) EdU assay was used to detect the proliferation ability (×200). (**C**) Scratch assay was used to detect the migration ability. (**D**) Transwell assay was used to detect the invasion ability (×200). (**E**) Western blot was used to detect the expression of fibrosis proteins. *, *P*<0.05, **, *P*<0.01, ***, *P*<0.001 compared with the siNC + INC group; ^##^, *P*<0.01, ^###^, *P*<0.001 compared with the siNC + miR-93-5p inhibitor group; ^&^, *P*<0.05, ^&&&^, *P*<0.001 compared with the siPVT1 + INC group. The data among multigroups were analyzed by one-way ANOVA, followed by Tukey’s test (between two groups).

RETRACTED

### Silencing of PVT1 blocked PI3K/Akt/mTOR pathway in HG-induced MMCs

The expression of PI3K/Akt/mTOR pathway related proteins was detected by Western blot. The expression of p-PI3K/PI3K, p-Akt/Akt, and p-mTOR/mTOR was higher in the siNC + miR-93-5p inhibitor group and was lower in the siPVT1 + INC group than that in the siNC + INC group (all *P*<0.001). The blocking effect of siPVT1 on PI3K/Akt/mTOR pathway was eliminated by miR-93-5p inhibitor (all *P*<0.001) (Figure 8).

**Figure 8:** LncRNA-PVT1 and miR-93-5p mediated the PI3K/Akt/mTOR pathway in MMCs under HG condition Western blot was used to detect the expression of PI3K/Akt/mTOR proteins (p-PI3K/PI3K, p-Akt/Akt, and p-mTOR/mTOR). ***, *P*<0.001 compared with the siNC + INC group; ^###^, *P*<0.001 compared with the siNC + miR-93-5p inhibitor group; ^&&&^, *P*<0.001 compared with the siPVT1 + INC group. The data among multigroups were analyzed by one-way ANOVA, followed by Tukey’s test (between two groups).

## Discussion

DN is one of the most common conditions found in patients with renal disease. Although PVT1 has been proved to be associated with DN, the detailed molecular mechanism of PVT1 in DN progression remains unclear. Here, PVT1 was found to be overexpressed in kidney tissues of ND mice and HG-induced MMCs. Silencing of PVT1 inhibited the proliferation, migration, invasion and fibrosis, promoted the apoptosis, and blocked PI3K/Akt/mTOR pathway in HG-induced MMCs. In addition, PVT1 negatively regulated its target miR-93-5p in MMCs. MiR-93-5p eliminated the effects of PVT1 on the biological processes of HG-induced MMCs.

Mesangial cells (MCs) are key functional cells in the development of DN, which can mediate the glomerular filtration rate [27]. Overproliferation of MCs is involved in the development of NC [28]. lncRNAs play important regulatory roles in the progression of DN. Gao et al. proved that lncRNA-ASncmtRNA-2 is up-regulated in DN kidney tissues and HG-treated MCs, and its overexpression promotes the glomerular fibrosis in DN [29]. Li et al. showed that lncRNA-1700020I14Rik contributes to the fibrosis of MMCs cultured with HG medium [30]. Wang et al. proved that overexpression of lncRNA-ENSMUST00000147869 reversed DN-induced proliferation and fibrosis of MCs [31]. The cell proliferation and fibrosis can also be regulated by lncRNA-CYP4B1-PS1-001 in DN [32]. Actually, as a member of lncRNAs, PVT1 also participates in the cell proliferation, migration, invasion, and fibrosis in diseases [33,34]. Huang et al. showed that PVT1 overexpression promotes the cell migration and invasion, and is a potential prognostic biomarker of small-cell lung cancer [35]. Zhao et al. proved that PVT1 promotes the migration and proliferation of pancreatic cancer cells via targeting miR-448 [34]. Alvarez et al. proved that PVT1 is up-regulated for five-folds in response to hyperglycemia, and PVT1 can mediate the accumulation of extracellular matrix in DN [16]. Here, PVT1 was up-regulated in DN kidney tissues and HG-induced MMCs. Silencing of PVT1 significantly inhibited the proliferation of HG-induced MMCs through blocking the cell cycle at G_0_/G_1_ phase, as well as the migration, invasion, and fibrosis of HG-induced MMCs. We speculate that PVT1 silencing may contribute to the remission of DN through mediating the above cellular biological processes.

RETRACTED

Some miRNAs mapping to the PVT1 locus play important roles in disease progression [36]. LncRNA-MEG3 inhibits the proliferation of glioma cells by targeting miR-93 and blocking PI3K/AKT pathway [37]. MiR-93 is a metabolic/epigenetic switch in diabetes, which connects the metabolic state and chromatin remodeling [38]. Zou et al. indicated that the plasma level of miR-93 was a potential predictor for high risk of diabetes-related diseases [39]. Furthermore, the regulatory pathway of PI3k/Akt/mTOR is important in the biological process of DN [40]. The phosphorylation of AKT and mTOR is a landmark reaction of DN [41]. Akt/mTOR pathway is a potential target to prevent renal fibrosis in DN [42]. MiR-196b and miR-451 influence the cell proliferation and invasion through regulating PI3K/AKT/mTOR pathway in cancer cells [43,44]. In this study, miR-93-5p inhibitor counteracted the inhibitory effect of siPVT1 on PI3K/Akt/mTOR pathway. We speculate that the PVT1 may activate the PI3K/Akt/mTOR pathway through targeting miR-93-5p, thereby regulating the proliferation, apoptosis, migration, invasion, and fibrosis of HG-induced MMCs. However, our findings are mainly performed on the biological processes of HG-induced MMCs. The regulatory effect of PVT1 in animal models of DN is still needed. The following assays in DN mice will be considered in our future researches: the kidney injury observed by HE staining, the levels of inflammatory factors detected by ELISA, and the activation of PI3K/Akt/mTOR pathway detected by Western blot.

RETRACTED

## Conclusions

Silencing of PVT1 inhibited the proliferation, migration, invasion and fibrosis, promoted the apoptosis, and blocked PI3K/Akt/mTOR pathway in HG-induced MMCs through targeting miR-93-5p. PVT1 was speculated as a potential therapeutic target for DN.

## Highlights

- PVT1 promoted proliferation, migration and invasion on HG cultured MMCs.
- PVT1 promoted fibrosis on HG cultured MMCs.
- The miR-93-5p as the target gene of LncRNA-PVT1.
- PVT1-miR-93-5p regulatory relation activated PI3K/Akt/mTOR pathway in DN.

## Abbreviations

DLR: dual-luciferase reporter
DN: diabetic nephropathy
ELISA: enzyme-linked immunosorbent assay
HE: hematoxylin eosin
HG: high glucose
HRP: horseradish peroxidase
INC: inhibitor negative control
miRNA/miR: microRNA
MMC: mouse mesangial cell
NC: negative control
PI: propidium iodide
PVT: lncRNA-plasmacytoma variant translocation 1
siPVT1: PVT1 siRNA
SPF: specific pathogen free
